The article "An Efficient Signal Processing Algorithm for Detecting Abnormalities in EEG Signal Using CNN" was published in 2022. Journal: Contrast Media Mol Imaging.

# An Efficient Signal Processing Algorithm for Detecting Abnormalities in EEG Signal Using CNN

**DOI:** 10.1155/2022/1502934

**Published:** 2022-09-21

**Authors:** Thalakola Syamsundararao, A. Selvarani, R. Rathi, N. Vini Antony Grace, D. Selvaraj, Khalid M. A. Almutairi, Wadi B. Alonazi, K. S. A. Priyan, Ramata Mosissa

**Affiliations:** ^1^Department of Computer Science and Engineering, Kallam Haranadha Reddy Institute of Technology (KHIT), Dasaripalem 522019, Andhra Pradesh, India; ^2^Department of Electronics and Communication Engineering, Panimalar Engineering Collage, Chennai 600123, Tamil Nadu, India; ^3^School of Information Technology and Engineering, Vellore Institute of Technology, Vellore 632014, Tamil Nadu, India; ^4^Department of Electronics and Communication Engineering, R.M.D. Engineering College, Kavaraipettai 601206, Tamil Nadu, India; ^5^Department of Electronics and Communication Engineering, Panimalar Engineering College, Chennai 600123, Tamil Nadu, India; ^6^Department of Community Health Sciences, College of Applied Medical Sciences, King Saud University, P. O. Box: 10219, Riyadh 11433, Saudi Arabia; ^7^Health Administration Department, College of Business Administration, King Saud University, PO Box: 71115, Riyadh 11587, Saudi Arabia; ^8^Department of Biotechnology, Sejong University, Seoul, Republic of Korea; ^9^Department of IT, Mettu University, Metu, Ethiopia

## Abstract

Electroencephalography (EEG) is crucial for epilepsy detection; however, detecting abnormalities takes experience and knowledge. The electroencephalogram (EEG) is a technology that measures brain motion and represents the brain's function. EEG is an effective instrument for deciphering the brain's complicated activity. The information contained in the EEG signal pertains to the electric functioning of the brain. Neurologists have typically used direct visual inspection to detect epileptogenic abnormalities. This method is time-consuming, restricted by technical artifacts, produces varying findings depending on the reader's level of experience, and is ineffective at detecting irregularities. As a result, developing automated algorithms for detecting anomalies in EEGs associated with epilepsy is critical. The construction of a novel class of convolutional neural networks (CNNs) for detecting aberrant waveforms and sensors in epilepsy EEGs is described in this research. In this study, EEG signals are analyzed using a convolutional neural network (CNN). For the automatic detection of abnormal and normal EEG indications, a novel deep one-dimensional convolutional neural network (1D CNN) model is suggested in this paper. The regular, pre-ictal, and seizure categories are detected using this approach. The proposed model achieves an accuracy of 85.48% and a reduced categorization error rate of 14.5%.

The article "An Efficient Signal Processing Algorithm for Detecting Abnormalities in EEG Signal Using CNN" was published in 2022. Journal: Contrast Media Mol Imaging.

## 1. Introduction

A disease is an anomalous problem that impacts an individual's body. A specific collection of clinical manifestations accompanies any deviations from the normal anatomy of a physical feature or function. The electroencephalogram has been used to identify illnesses of the brain. The monitoring of neuronal activity from such a skull is known as an electroencephalogram [1]. It monitors the voltage changes caused by ionic current that starts flowing in the brain or spinal cord. The spectrum content of EEG, or the type of brain oscillation that can be seen in EEG data, is usually the target of medical diagnostics. EEG is noninvasive and painless. It also does not allow any electrical to enter your brain or body. Omega, delta, beta, gamma, and alpha are five EEG sub-bands that are often dissected. Alpha waves have a frequency spectrum of 8 to 13Hz and thus are repetitive. The alpha waveform has small amplitude [2]. The alpha frequency can be found in any part of the brain; however, it is most commonly recorded in the occipital and parietal areas. It alternates between an awakened adult and a comfortable person with closed eyelids.

Beta waves have a frequency spectrum of more than 13 Hz and are irregular. The beta waveform has relatively small amplitude. The temporal and frontal lobes are where it is usually reported. It is linked to memorizing and vibrates between profound sleep, brain functions, and memory. Delta waves have a frequency spectrum of 4 to 7 Hz and are continuous. The delta waveform has large amplitude. The occipital lobe fluctuates between sleepy youngsters, drowsy adults, and emotional anguish [3]. Theta waves have a frequency spectrum of less than 3.5 Hz and are sluggish. Theta waves have a low-medium frequency. It alternates between an adult and a regular sleep schedule. The quickest brainwave wavelength is gamma impulses, which have a frequency spectrum of 31 to 100 Hz as well as the shortest intensity. The EEG inputs are converted into the preprocessing system. The discrete wavelet transform is employed to remove disturbances from the preprocessing, and the EEG signal is separated into five sub-band signals [4]. Each one of the six EEG signals had its nonlinear properties (time and frequency) removed. The best characteristics from the retrieved time and spatial frequency characteristics were extracted using a genetic algorithm. The classification can then be used to determine whether the EEG signal is healthy or unhealthy.

Unrestrained electrical discharges in such a network of neurons lead to seizures. Brain function is affected as a result of an abnormal emission of electrons. When at least two spontaneous seizures occur in a row, epilepsy is established. It can impact people of all ages. Patients must receive a complete and rapid diagnosis of epilepsy, which is needed to commence antiepileptic drug treatment and, as a result, lower the risk of future seizures and seizure-related problems. Taking a complete timeline, doing a neurological assessment, and taking supplementary tests such as neuroimaging and EEG are currently used to diagnose epilepsy [5]. Inter-ictal (among seizures) and epileptic (throughout a seizure) epileptogenic anomalies can be detected using EEG signals. However, visualization of data of EEG signals is time-consuming, especially with a rising usage of the outpatient mobility EEGs and inpatient video stream EEG records, when hours to several days amount of EEG data must be visually evaluated. Although most EEG software contains a variety of electronic automatic detection, current methods of automation detection and diagnosis are hardly employed in clinical practice due to the terrible specificity and sensitivity of the predetermined seizure recognition techniques.

The article "An Efficient Signal Processing Algorithm for Detecting Abnormalities in EEG Signal Using CNN" was published in 2022. Journal: Contrast Media Mol Imaging.

Furthermore, because of the fundamental nature of visual examination, clinical diagnoses differ depending on the EEG specialist's degree of proficiency in electroencephalography. To make matters more complicated, the study's integrity might well be harmed by conflicting artifactual signals, which impair the reader's capacity to precisely identify irregularities [6]. Aside from that, the low interest in routine outpatient investigations is an issue. An outpatient EEG can be performed on a patient with epilepsy, as well as the results may be perfectly normal. This is because epileptic individuals' brains are not constantly firing off epilepsy impulses. An EEG is an “image” of the brain taken at a time of soundtrack. The responsiveness of detecting epileptic releases could be enhanced by incorporating the patient return for repetitive inpatient research or capturing them for the longer time, either through household ambulant research or an inpatient audiovisual stream EEG monitoring research, and both are expensive and time-consuming for the client and the therapist trying to read an EEG.

The frequencies, intensity, and reflectivity on the scalp of EEG waves can all be characterized. During the classification stage, the signal's class (healthy or unhealthy) must first be identified. After that, by splitting the aberrant impulses into subcategories, the kind of neurologic illness can be determined. Seizures are conditions in which the electrical activity among neurons occurs in an aberrant manner as a result of abnormal EEG data. A generalized seizure occurs when a brain disorder extends to all areas of the brain [7]. A focused or partial seizure happens when the seizure only affects a few areas of the brain. Bioelectrical artifacts must be deliberately avoided during the recording of EEG signals by evaluating the seizures with numerous compilations to prevent unwanted and erroneous interpretation. The distinction between epileptic and nonepileptic convulsions aids in the identification of serious disorders like epilepsy [8]. Seizures may not always happen, and normal EEG signals are defined as those that are free of uncommon seizures. Because seizures identification is the first step in detecting aberrant brain functioning, numerous research articles are devoted to seizures identification and predictions.

The article "An Efficient Signal Processing Algorithm for Detecting Abnormalities in EEG Signal Using CNN" was published in 2022. Journal: Contrast Media Mol Imaging.

The slight differences in the voltage instability of the EEG recordings indicate that neural activity is occurring. As a result, the visual assessment of these indicators differs depending on the level of knowledge. Furthermore, manual analysis of extensive EEG recordings takes a very long time, and the conclusions can be erroneous due to the existence of artifacts in the signals. As a consequence, machine technologies can be used to analyze and examine these messages to provide quick and precise findings [9]. The use of computer-aided systems with EEG signals has grown in popularity, particularly, in the prediction of diseases, major depressing disorder (MDD), alcohol utilization disorder (AUD), and brain disorders such as Alzheimer's disease, minor cerebral impairment (MCI), Parkinson's disease, and dementia with Lewy bodies (DLB). The request of motor imagery based on EEG has opened up a novel door in the realm of neuroprocessing. Other study topics using physiological data such as EEG include identity identification, sleep phase categorization, facial emotion, eye state identification, and sleepiness tracking.

A preprocessing stage, extraction of features, and categorization are the most frequent sequential processes in the development of an automated detection method. Normalization and different transformations are obtained from the original signals in the preprocessing stage to normalize the pattern for subsequent stages. The unique characteristics included in the waveforms are recovered utilizing various approaches in the feature extraction phase. Hilbert–Huang transform, wavelet analysis, spectra features, and higher-order cumulate and principal components are some of the most often used feature representations. For the categorization of features generated via customized feature extraction methods, neural networks and support vector machines are commonly utilized. The evaluation is done using single and multiple observations [10]. EEG signals are complicated and nonlinear, necessitating the implementation of increasingly inventive machine learning and signal processing algorithms to analyze them. Recent breakthroughs in deep learning methodology have yielded potential methods for extracting complicated data characteristics at high degrees of abstraction automatically. These deep learning techniques have already been used in image processing, NLP, voice recognition, and computer gaming with great success. These algorithms have also been applied in the field of biomedicine. For the categorization of regular, pre-ictal, and seizure EEG signals, a 13-layer deep convolutional neural network (CNN) was developed. They achieved an 88.67 percent categorization rate, utilizing 300 EEG samples from five individuals in their investigation. Using a deep neural network technique, the same researchers suggested a unique EEG-based depressive screening program [11]. The efficiency scores for 15 normal and 15 depressed individuals were 93.5% (left hemispheres) and 96% (right hemisphere), respectively. Another research used EEG signals to offer a deep learning strategy for detecting Parkinson's illness. With a 13-layer CNN model created utilizing 20 healthy and 20 Parkinson's disease participants, they were able to attain an efficiency of 88.25%.

The article "An Efficient Signal Processing Algorithm for Detecting Abnormalities in EEG Signal Using CNN" was published in 2022. Journal: Contrast Media Mol Imaging.

The automatic detection of normal and pathological EEG signals is proposed in this paper using a deep learning-based method. Rather than using the manual feature extraction technique, a 23-layer comprehensive final 1D-CNN-based representation is specified [12]. From 1-minute chunks of EEG recordings, abnormal EEG signals were immediately recognized. The project's objectives are to detect unusual EEG for the treatment of nervous illnesses and to apply deep learning techniques to neuroscience utilizing a large EEG data set. The rationale stems from the fact that professional physical evaluation of EEG signals is taxing and time-intense, and that machine learning techniques can increase detection performance. A novel 1D CNN model was established for this objective and used for the first period on the EEG quantity subdatabase to accomplish this goal. Another noteworthy accomplishment was the effective use of only-channel 1-minute EEG segments rather than multichannel generated sections. Moreover, the recognition assignment in this research does not involve a brain image, which is advantageous for clinical analysis [13]. The remainder of the work is arranged in the following manner: the fundamentals, techniques, and suggested 1D CNN model are all introduced in Section 1; Section 2 explains the previous papers related to the study; Section 3 describes the experimental setting; Section 4 explains the proposed model, and the suggested model's effectiveness is presented in Section 5; Section 6 presents a commentary derived from the findings of Section 5; and eventually, the conclusion of this paper is presented in Section 7.

The article "An Efficient Signal Processing Algorithm for Detecting Abnormalities in EEG Signal Using CNN" was published in 2022. Journal: Contrast Media Mol Imaging.

## 2. Related Work

A new technique for diagnosing Parkinson's disease (PD) from the electroencephalogram (EEG) signals obtained from normal and PD-affected participants was developed and evaluated. In the assessment of EEG signals, the technique depends on sample entropy (SampEn), discrete wavelet transform (DWT), and three-way decision structure. Because the EEG signal is chaotic and nonstationary, it is hard to know visually. The system is a well-established three-stage paradigm for EEG signal processing. The DWT was used to obtain split frequency components in the first phase; in this phase, a three-level DWT was utilized to divide the EEG signal into the estimate and a detailed parameter; and then attempts were taken to remove worthless and noise data and obtain appropriate data. Approximation coefficients were used to generate the SampEn numbers in the next phase since SampEn has an advantage in assessing the EEG data. Finally, a three-way judgment based on the optimal center constructive covering algorithm (O-CCA) was used to detect PD patients with an accuracy of 92.86%. The detection rate drops to 88.10% when the DWT is used as a preprocessing stage. Overall, the suggested combination approach is acceptable and efficient for evaluating the EEG signal with more precision [14].

The most crucial physiological mechanism in human health is sleep. People's lives have been accelerated by societal growth, which has also raised their life pressures. As a result, a rising number of people are experiencing poor sleep quality, and the disorders that arise are also on the rise. In approach to this issue, this research presents an electroencephalogram-based technique for detecting and managing sleep excellence (EEG). The major method for sensing sleep excellence is to process sleep EEG data. Wavelet packet decomposition (WPD) synthesizes the unique EEG data to obtain the four EEG rhythm waves. Then, each rhythm wave's average energy parameters and nonlinear features are retrieved. The major features are the multisampling entropy (MSE) values of the dissimilar scales, while the remainder is supplementary features. Finally, the collected sleep characteristics are determined using the long short-term memory (LSTM) technique and the outcome is achieved. Investigations were performed on the shared database of the MIT-BIH. The results of the experiments suggest that the technique utilized in this paper has the highest accuracy for detecting sleep value. The data are maintained in conjunction with the mobile networking software for the discovered sleep accurate information. Management can be divided into two categories: the first is to run a query and see previous data on the quality of sleep; and the second would be that the customer would be alerted if there are periodic irregularities in an observed quality of sleep data, such that the user may react in time to maintain fitness levels [15].

The article "An Efficient Signal Processing Algorithm for Detecting Abnormalities in EEG Signal Using CNN" was published in 2022. Journal: Contrast Media Mol Imaging.

Depression is now a huge medical issue and financial impact all across the world. Due to the limits of present approaches for diagnosing sadness, a comprehensive and objective methodology is needed. A psychophysiological database encompassing 213 participants was created for this study. The electroencephalogram (EEG) signals of all subjects were obtained at *Fp*1, *Fp*2, and*Fpz* electrode sites during rest and sound activation using a widespread frontal cortex three-electrode EEG device. A total of 270 linear and nonlinear characteristics were retrieved after denoising with the finite impulse response filtering, which combined the Kalman derivation method, discrete wavelet transforming, and an adaptive estimator filter. The information space's dimensions were then decreased using the minimal-redundancy-maximal-relevance feature selection algorithm. The depressive respondents were discriminated from normal controls using four classification approaches (SVM, K-NN, decision trees, and ANN). The performance of the classifiers was assessed using 10-fold cross-validation. K-nearest neighbor (KNN) has the best accuracy of 79.27%, according to the data. The findings also revealed that the ultimate power of a theta waveform could be a useful indicator of depression. The viability of a widespread three-electrode EEG data acquisition unit for the diagnosable disorder is demonstrated in this work [16].

The categorization of seizures requires the identification of recorded epileptic neurological issues in electroencephalogram (EEG) portions. Manual identification is a time-consuming and arduous technique that builds a significant strain on neuroscientists; hence, automated epilepsy detection has become a major concern. Current EEG detection systems rely heavily on artificial knowledge and have a limited ability to generalize. This presents a unique one-dimensional deep neural network for the robust automatic recognition that consists of three convolutional blocks fully connected to overcome these constraints. Each convolution blocks have five layers: a max-pooling surface, a convolutional neural network, a batch normalization layer, a dropout layer, and a nonlinear activation surface. The accuracy of the system is tested using the University of Bonn data set, which obtains 97.63% in a two-class classification task, 96.72% in a three-class EEG categorization challenge, and 93.55% in categorizing the complex five-class issues [17].

The article "An Efficient Signal Processing Algorithm for Detecting Abnormalities in EEG Signal Using CNN" was published in 2022. Journal: Contrast Media Mol Imaging.

Epilepsy is a nervous system illness caused by massive brain cell activity. Recurrent spontaneous seizures are the most common symptom. Electroencephalogram (EEG) signals can be utilized to identify and analyze this neurological disorder. Many methods have been used to obtain good performance in the epileptic EEG categorization. The intricacy and unpredictability of EEG signals make it difficult for researchers to apply the necessary algorithms. Sample complexity on multidistance signaling level difference (MSLD) was utilized in this research to determine the characteristics of EEG signals, particularly in epilepsy-affected people. The test was conducted on three types of EEG data: ictal (seizure) impulses from epilepsy patients, ictal (nonseizure) information from healthy participants, and ordinary EEG signals from healthy people with closed eyes. The support vector machine (SVM) approach was used to categorize and verify the data in this investigation. Experiment findings indicated the maximum accuracy of 97.7% using 5-fold cross-validation [18].

## 3. Materials and Method

### 3.1. EEG Signal Processing Analysis

In this research, a deep convolutional neural network approach was utilized to categorize healthy and unhealthy EEG signals. This framework allows the impulse to be entirely predictable in an end-to-end circuit without requiring a feature extraction process.  Figure 1 depicts the phases needed in the automatic recognition of abnormal EEG readings:

1. Preprocessing stage
2. Extraction of features
3. Feature selection
4. Classification process

The EEG signal preprocessing approach is covered in the first module. It is used to filter out noise from such a signal [19]. The EEG signal features are extracted from the fragmented signal in the next component. Then, from the retrieved features, the appropriate features are chosen. The categorization method uses the selected features as parameters. The categorization method is mostly used to analyze EEG signals and divide them into physiologic and pathologic categories.

The modest fluctuations in EEG measurements efficiently reflect the brain's continually shifting functioning states. Furthermore, the EEG of a normal person differentiates from that of an abnormal person [20]. As a result, it is critical to recognize those changes using a variety of signal collection and analysis processes, as well as computer-assisted techniques. Preprocessing, extraction of features, postprocessing, and outcome analysis are the four processes. The raw data could be directly supplied to the results evaluation stage for categorization or statistical methods, namely, any of the first three stages of the treatment process could be bypassed depending on the design, as shown in Figure 1. Feature selection or extraction of features is not needed to be undertaken individually in certain research investigations where deep neural networks have been used for data processing [21]. If the information has been previously preprocessed or the characteristics have already been identified, either of those processes can be avoided. This is especially true for standard data sets. Again, if the retrieved feature set is tiny, no postprocessing with selecting features or matrix factorization approaches is required. Finally, during the results analysis process, categorization or statistics analysis was conducted with the goal of detecting some abnormality or recognizing various functioning stages of a brain in order to track certain applications.

The article "An Efficient Signal Processing Algorithm for Detecting Abnormalities in EEG Signal Using CNN" was published in 2022. Journal: Contrast Media Mol Imaging.

## 4. Proposed Methodology

A deep convolutional neural network method is established to categorize healthy and unhealthy EEG signals in this research. Without any feature extraction phase, this framework enables the impulses to be completely standard in an end-to-end comprehensive construction [5]. The stages in the automatic identification of an aberrant EEG signals are depicted in Figure 2.

The goal of producing the data sets is to give adequate scientific evidence for a creation of information-driven tools and to establish an essential point. The most useful feature of such a data set is that each EEG signal comes with a report from the physician. The clinical description of the patients and a description of the drug are included in these data sets [22]. The TUH aberrant EEG Corpora (*v*2.0.0) database, which contains both normal and pathological EEG signals, is used in this work. The signals are divided into two categories: training and evaluation. The number of participants and events used in the TUH EEG Irregular Corpus (*v*2.0.0) data set is shown in Table 1. Even during training and estimation sets, there is no clinical disagreement. The only patient information either regular or irregular is being used in the assessment database. During training, just a few patient records appear numerous times. In conclusion, the assessment data set has 253 different individuals, while the training data set contains 2076 distinct patients. Each patient may have more than a session.  Table 2 represents the frequency of patients in the EEG data set.

The article "An Efficient Signal Processing Algorithm for Detecting Abnormalities in EEG Signal Using CNN" was published in 2022. Journal: Contrast Media Mol Imaging.

Information from 24 to 36 channels is present in the EEG system database, and streams are labeled with important event indicators. The EEG information was verified at a sampling degree of 250 Hz and a resolution of 16 bits per sample. The positions of the channels sensors used to obtain the accounts are shown on the left sideways of Figure 3, while the first 60-s signal patterns of the anomalous highest are shown on the correct side [23]. A conventional EEG system comprises a 19-electrode layout, although extra sensors can be added to improve the amount of spatial data obtained.

## 5. Convolutional Neural Network (CNN)

In this study, a newly designed and upgraded neural network known as the convolutional neural network (CNN) is used. Shift and translational invariance are both enhanced in the ANN. The CNN's convolution layer is a subclass of deep learning that has gotten a lot of buzz in new times and is utilized in image processing applications, including X-ray medical images, histopathological pictures, magnetic resonance imaging, fundus images, and computed tomography pictures [24]. However, there seems to be little study on the application of CNN with physiological data. Thus, in prior work by researchers, the CNN has been used to analyze ECG signals to determine the usefulness of the CNN process in signal processing. Using varied periods of tachycardia ECG sections, the CNN was used to automatically identify arrhythmia with an accuracy rate of 92.5% and 94.9% using 2-second and 5-second ECG portions, respectively. The use of CNN in the automatic identification of myocardial injury, peripheral arterial disease, and categorization of various heartbeats utilizing ECG signals was recently revealed.

The CNN model, like the ANN, bases its final feature selection on the connection weights of previous levels in the underlying network. As a result, for each layer, equations (1) and (2) are used to modify the model's weights and biases.

(1) $$\begin{array}{c} {∆W}_{e}\left(t+1\right)=-\frac{x\lambda }{k}W_{e}-\frac{a}{n}\frac{\partial C}{\partial W_{e}}+m{∆W}_{e}\left(t\right), \end{array}$$

(2) $$\begin{array}{c} {∆B}_{e}\left(t+1\right)=-\frac{a}{n}\frac{\partial C}{\partial W_{e}}+m{∆B}_{e}\left(t\right). \end{array}$$

Here, the weight, biases, layer amount, regularization variable, rate of learning, the overall amount of training data, energy, update stage, and cost function are represented as *W*, *B*, *e*, *λ*, *a*, *n*, *m*, *t*, an d *C*, respectively

Regularization, rate of learning, and velocity are the variables required for training the CNN model. To obtain optimum performance, these variables can be modified according to the data set. The lambda is used to avoid data fitting problems. The training error determines how quickly the network understands during training, whereas velocity aids in data converge. In this work, the variables lambda, rate of learning, and velocity are set at 0.7, 1 × 10^−3^, and 0.3, respectively. These values were discovered through experimental and fault error [25]. This study is the initial application of CNN for the EEG signal analysis in overall and appropriation identification specifically, to the authors' knowledge. The convolutional layer, pooling layer, and fully connected layer make up the CNN model.

The article "An Efficient Signal Processing Algorithm for Detecting Abnormalities in EEG Signal Using CNN" was published in 2022. Journal: Contrast Media Mol Imaging.

### 5.1. Convolutional Layer

Filters (kernels) slide throughout the EEG signal in this system. The kernels are the matrices that will be combined also with the input of EEG signal, while the step determines the filtering will characterize over the signal. This layer employs the kernel to conduct multiplication on the given EEG signals. The convolution layer is another name for the convolution's outputs. Equation (3) is the convolution procedure:

(3) $$\begin{array}{c} b_{k}=\overset{N-1}{\underset{n=0}{\sum }}a_{n}r_{k-n}, \end{array}$$

where *a* represents the signal, *r* represents the filter, and *N* is a quantity of fundamentals in *a*. *b* is the output path. The *n*th component of the vector is denoted by the constants.

### 5.2. Pooling Layer

The downsampling level is another name for this layer. To reduce the computation complexity and minimize generalization error, the pooling process will reduce the number of output nodes from the convolution layers. In this paper, the max-pooling technique is utilized. The max-pooling process chooses only its maximum priority in every convolution layer, resulting in fewer output nodes.

### 5.3. Fully Connected Layer

In this research, the activation function consists of two types: (a) soft-max layer and (b) rectified linear activation unit.

### 5.4. Soft-Max Layer

The posterior distribution of a *k* output class is computed using this method. As a result, Layer 13 employs the soft-max activation function to determine whether the class that input EEG signals corresponds to (regular, pre-ictal, or seizures).

(4) $$\begin{array}{c} p_{j}=\frac{e^{a_{j}}}{\sum_{1}^{k}e^{a_{k}}}\;for\;j=1,\ldots k. \end{array}$$

Here, the total input is denoted by *a*. The output range of *p* is from 0 to 1, and its total equals 1.

### 5.5. The Rectified Linear Activation Unit

It is usual practice to use an activation function after each convolutional layer. An activation function is a procedure for mapping output to a set of input data. They are employed to give the communication network nonlinearity. The rectifier linear unit is a well-known deep learning scale parameter. As a convolution operation for the convolutional layers, the leaky rectified linear unit (Leaky-ReLU) is being used in this study. The features of a Leaky-ReLU contribute nonlinearity and sparseness to the system structure. As a result, giving stability to tiny changes in the input, including noise, the Leaky-ReLU functional is shown in

(5) $$\begin{array}{c} f\left(a\right)=\left\{\begin{array}{c} a\;if\;a>0,\\ 0.01a\;otherwise. \end{array}\right) \end{array}$$

The article "An Efficient Signal Processing Algorithm for Detecting Abnormalities in EEG Signal Using CNN" was published in 2022. Journal: Contrast Media Mol Imaging.

### 5.6. 1-Dimensional CNN Model

For the automatic analysis of regular and irregular EEGs, a unique 1-dimensional convolutional neural network model has been developed. The input layer is one of 23 levels in the planned deep network architecture. 1D convolutional layer, max-pooling, dropout layer, batch normalization, and dense layers are all included in the constructed model. The deep learning 1D CNN model is presented in Figure 4. The model's first layer is composed of real EEG signals. The CNN model that follows after the input layer requires four-step periods and eight filtering with 23 elements to conduct a combination on the original signal [26]. Extracted features of the carrier frequency are formed after the convolution process. Two-unit regions on such extracted features are decreased in the max-pooling phase to the optimum amount in these areas.

Based on the size of pooling and pace parameters, the area of the feature maps is reduced by approximately. Regularization is one of the most difficult problems in deep architecture. Dropout has been the most popular method for preventing overfitting. Dropout layers are included in different positions in the suggested deep model to prevent it from overfitting. In each group, the batch normalization layers are utilized to regularize the inputs of the preceding layer [27]. Also with the conversion approach, the theory indicates a near-zero activating median and a near-one initiation confidence interval throughout batch normalization. The thick layers have such a neural network topology that is highly coupled. The flattening layer undergoes dimension modifications, so that the attributes of the preceding layer can be treated in fully connected layers. The soft-max layer, which executes the categorization, is the model's final layer. The input EEG data is categorized as healthy or unhealthy in this layer. The features and parameters utilized in a suggested 1D CNN model are shown in Figure 4.

The system has a total of 382,682 characteristics, 382,634 of those are trainable and 48 of those are nontrainable. The 1D convolution entire image is represented by the kernel designed product. During the model's designing phase, overfitting is the most common issue. After many modifications to the quantity of hidden layers and the hyperparameters, a best model was found. The quantity of hidden layers in the 1D CNN model and the characteristics of these levels are determined using the brute force method. Optimal layers and parameter tweaks are done regularly after verification to provide better results.

The article "An Efficient Signal Processing Algorithm for Detecting Abnormalities in EEG Signal Using CNN" was published in 2022. Journal: Contrast Media Mol Imaging.

### 5.7. CNN Model Training

In this study, the CNN is trained using traditional backpropagation (BP) with a total sample size of three. BP is a way of calculating the loss function's gradient with appropriate weights. While training, BP sends error signals backward across the system for such parameters to be modified. The number of signals used in each training session is referred to as the sample size. In this project, factors related to three are used.

### 5.8. CNN Testing Model

In this study, 150 training iterations were completed. One cycle of the whole training set is denoted as iteration. This approach evaluates the CNN model with each cycle of an epoch while using 30% of the overall training data set (70%) to validate the model. The pattern among all the EEG signals used for this study is depicted in Figure 5.

### 5.9. K-Fold Cross-Validation

This research used a 10-fold cross-validation technique. To begin, the EEG data are separated into ten equal amounts at randomness. 9 out of 10 segments of EEG data were utilized to training the CNN, although the other one-tenth is used to test the network efficiency [28]. By swapping the testing and training data sets ten times, this process is repeated. The results for precision, sensitivity, and selectivity provided in this report are the averages of ten assessments.

## 6. Results and Discussion

In this research, a deep learning framework for automatically classifying normal and pathological EEG signals was built. This database's information is divided into two categories: training and evaluation. These statistics are calculated to train and test the model during the experimental research. This study's experimental setting suggested that the first 60 seconds of EEG records be used. The signals collected from 24 to 36 separate channels are stored in the EEG information in the database. In both, only subsequent temporal to occipital (T5–O1) and right frontal to central (F4–C4) channel impulses were employed. The T5–O1 divergence observation, which would be part of the mainstream temporal central parasagittal (TCP) composite, has been the most probable channel for manual interpretation. For reference, the F4–C4 channel signals were analyzed. In the TCP construction, Figure 6 depicts the graphical presentation of T5–O1 an d F4–C4 EEG signals. The first 60 seconds of each EEG recording have been used in this research. Each one of these sections has 15,000 observations, which were given into the CNN model provided input. The signals have not been subjected to any manual feature extraction. The signals were normalized to 0–1 during the preprocessing stage and then identical by eliminating the average and scaled to unit modification. The first 60 seconds are usual and aberrant T5–O1 channel EEG recordings.  Table 3 lists the most important hyperparameters for use in CNN architecture implementation.

The article "An Efficient Signal Processing Algorithm for Detecting Abnormalities in EEG Signal Using CNN" was published in 2022. Journal: Contrast Media Mol Imaging.

The EEG signals were taken from the TUH-EEG data set. The recordings in the EEG database were divided into two categories: training phase and evaluation phase. During the stage of learning, the training data set has been used, but during the testing phase, evaluation data set has been used. The CNN classifier is constructed using 80% of the training examples, while the other 20% is used as a validation set. Thus, 2173 data out of several 2717 are being used for training, and 544 records have been used for validation. These data ranges were chosen at random. The T5–O1 pathway, which is generally recognized by specialists, yielded the results of the experiment.  Figure 7 displays the effectiveness graphs of the CNN model for this channel even during the training stage for 150 iterations; and the blue curve indicates the training set and the orange curve indicates the validation set in Figure 7.

The effectiveness graphs show that the model does not have an overfitting problem. The training performance of the results is in the region of 78–79 percent, and the validating prediction accuracy is also in the range of 79–80 percent. The training loss value, which had previously been 0.78, has now dropped to 0.46. Given the difficult data, the model was unable to complete the preprocessing step.

Experimentation with various hyperparameters has revealed problems with over fluctuations and generalization error during the training and testing data phases and after the system has completed the training phase. Another significant routine breakthrough of a trained CNN model is its ability to perform well with testing data not encountered during the training process. Different assessment parameters for the testing data set have been chosen for this aim. Accuracy, precision, recall, and *F*1-score were the parameters used to compare the efficiency of the proposed method. True positive, true negative, false positive, and false negative are represented as (*T*_*postive*_), (*T*_*Negative*_), (*F*_*positive*_), and (*F*_*Negative*_), respectively.

The article "An Efficient Signal Processing Algorithm for Detecting Abnormalities in EEG Signal Using CNN" was published in 2022. Journal: Contrast Media Mol Imaging.

### 6.1. Accuracy

Accuracy is the quantity of accurately calculated facts separated by the overall number of observed. It is a commonly used evaluation criterion, and the formula for calculating is given in

(6) $$\begin{array}{c} accuracy\left(\%\right)=\frac{T_{positive}+T_{negative}}{T_{positive}+T_{negative}+F_{positive}+F_{negative}}. \end{array}$$

### 6.2. Precision

Precision is the ratio of accurately assessed positive events to a total number of assessed positives. Equation (7) can be used to assess it.

(7) $$\begin{array}{c} Precision\left(\%\right)=\frac{E}{T_{positive}+F_{positive}}\times 100. \end{array}$$

### 6.3. Recall

Recall is the percentage of appropriately identified explanations in a class compared to the total number of observations within this class. Sensitivity is another term for recall, which is calculated using

(8) $$\begin{array}{c} recall\left(\%\right)=\frac{T_{positive}}{T_{positive}+T_{negative}}\times 100\text{.} \end{array}$$

### 6.4. *F*1-Score

It is a subjective mean of exactness and memory. Equation (9) can be used to determine it.

(9) $$\begin{array}{c} F1-score=\frac{\left(recall\right)\times \left(precision\right)\times 2}{\left(recall\right)+\left(precision\right)}. \end{array}$$

Using 276 sessions, the constructed model by using the T5–O1 signal is assessed. The different performance measurements derived for the constructed model are presented in Table 4. The test EEG signals were identified by the constructed CNN model with the highest accuracy ratio of 85.48 percent and a recall value of 78.72 percent.

Thus, the effectiveness of the algorithm using EEG signals from the F4–C4 channels without modifying any set of parameters is tested.  Figure 8 depicts the generated model's effectiveness graphs using F4–C4 channel EEG signals across 152 training iterations; and the blue curve indicates the training set and the orange curve indicates the validation set. The overfitting issue did not emerge even during the training process for the system developed utilizing F4–C4 channel EEG data, and the validating prediction accuracy was 74 *to* 81%. The prediction error, which was 14.5% throughout the model's training, dropped to 0.19% after 150 iterations. 279 test data were given into the model that had been trained on F4–C4 EEG channel data. The different performance metrics collected for the constructed model are presented in Table 4.

The assessment EEG signals were categorized from the F4–C4 channel using the constructed CNN model, which had an overall accuracy percentage of 80.65% and a recall rate of 78.2%.  Table 5 shows the performance comparison between the proposed and existing models. With an accuracy of 75.64%, the suggested model accurately identified 136 of 150 F4–C4 channel EEG data. The model performed slightly worse when it came to recognizing aberrant EEG data.

The article "An Efficient Signal Processing Algorithm for Detecting Abnormalities in EEG Signal Using CNN" was published in 2022. Journal: Contrast Media Mol Imaging.

The findings reveal that throughout both the training and testing stages, the generated model significantly outperformed with T5–O1 channel on EEG data than with F4–C4 channels EEG information. For both channels' EEG readings, the model's hyperparameters were left unchanged.  Figure 9 depicts the effectiveness of the constructed model utilizing EEG signals from the T5–O1 and F4–C4 channels during a training period; and the blue curve indicates the training set and the orange curve indicates the validation set.

In this research, a 1D CNN model is employed to categorize usual and unusual EEGs using the TUH-EEG aberrant data set. In their investigation, they used a 0.1 s frame length for extraction of features on the first 60 s images of T5–O1 channel signals.

The proposed method correctly categorized EEG data with a reduced 14.5% error rate using CNN. For the detection of aberrant EEG signals, the researchers employed four-channel EEG signals for a 7-s frame length of the first 60 s period. Also, with the 2*D*CNN model, they obtained a 21.2% failure rate for the occipital area. On the EEG signals, mainly initial normalization and standardization operations are done in this investigation. In this investigation, the first 60 seconds (15,000 samples) of the T5–O1 channel EEG data were used. With an error rate of 20.6%, the proposed 1D CNN model automatically distinguishes healthy and unhealthy recordings. Aside from extracting the features, the 1D CNN model offers additional benefits including the retrieval of 1D subsets from the data with limited features and preprocessing within the convolutional layer. Because of these benefits, the 1D CNN model is well suited to single-channel EEG signal structures.

Table 5 shows the comparison of existing and proposed mechanism to validate the efficiency of the proposed mechanism. It shows that the proposed mechanism out performs the existing mechanism in terms of various parameters like accuracy, precision, recall, and *F*1-score with the value of 85.48%, 76.65%, 78.2%, and 69.12%, respectively.  Figure 10 shows the graphical representation of comparison representing the efficiency of the proposed method with other methods.

An experiment is carried out in this study using access to the TUH EEG abnormalities dataset without modifying the experimental system. In future investigations, we plan to analyze information over a longer time and also propose employing multichannel EEG neural impulses to do categorization. Only the first 60 seconds of each EEG record were used as data input in this investigation. The lengths of the segments should be reduced to increase the quantity of collected data. Additional deep learning methods, including LSTM, CNN-LSTM, and CNN-LSTM, can be used to increase classification performance in addition to a CNN algorithm.

The article "An Efficient Signal Processing Algorithm for Detecting Abnormalities in EEG Signal Using CNN" was published in 2022. Journal: Contrast Media Mol Imaging.

## 7. Conclusion

The analysis of EEG signals to detect brain disorders is a complex task. As a result, for the diagnosis of brain disorders, a PC-based automatic system is required. This research could be valuable in the study of both healthy and unhealthy patients. This article presents a 1D-CNN-based technique for an automatic recognition of aberrant EEG signals. According to the research, each stage plays a critical role in the extraction of raw EEG signals. Preprocessing, extraction of features, postprocessing, and outcome analysis were all significant stages in transforming raw time domain of EEG signals for constructing automated evaluation methods. The proposed work assists in early diagnosis of aberrant EEG signals with an accuracy of 85.48%, a precision rate of 76.65%, and a reduced error rate of 14.5%. The comparison shows that the proposed method outperforms the existing work with increased accuracy and reduced error rate. Thus, in future, the plan is to increase the efficiency by combining the optimization mechanism with the deep learning methods to enhance the efficiency.

## Figures and Tables

**Figure 1:** Framework for EEG signal analysis.

**Figure 2:** Steps for automatic detection of abnormal EEG signals.

**Figure 3:** A graphical representation of the EEG sensor locations.

**Figure 4:** Block diagram of the 1D CNN structure.

**Figure 5:** Distribution of EEG data utilized in the suggested algorithm's testing and training.

**Figure 6:** T5 − O1 an d F4 − C4 EEG signal graphical representation.

**Figure 7:** T5–O1 EEG signal data: (a) accuracy model and (b) loss model performance during the training stage.

**Figure 8:** F4–C4 EEG signal data: (a) accuracy model and (b) loss model performance during the training stage.

**Figure 9:** Level of training using T5–O1 and F4–C4 EEG signal channel.

**Figure 10:** Performance comparisons of existing and proposed methods.

**Table 1:** Description values of affected role and assembly in TUH-EEG.

Parameter	Affected role			Assembly		
	Healthy	Unhealthy	Overall	Healthy	Unhealthy	Overall
Training	1238	894	2132	1370	1349	2719
Evaluation	149	106	255	152	127	279
Overall	1387	997	2384	1522	1473	2995

**Table 2:** Patient gender ratio in the EEG given data set.

Parameter	Training data set		Evaluation data set	
	Patients	Files	Patients	Files
Female (regular)	690	765	85	86
Female (irregular)	456	680	52	64
Male (regular)	545	605	65	67
Male (irregular)	438	676	53	64
Overall	2129	2726	255	281

The article "An Efficient Signal Processing Algorithm for Detecting Abnormalities in EEG Signal Using CNN" was published in 2022. Journal: Contrast Media Mol Imaging.

**Table 3:** Values for the deep 1D CNN model.

Number	Elements	Standard values
1	Optimization	A da m, beta 1=0.8 an d beta 2=0.99
2	Rate of learning	0.00001
3	Error function	Cross categorical entropy
4	Iterations	150
5	Decay	1*e* − 3
6	Size of batch	127
7	Metrics	Precision

**Table 4:** Performance estimates of the model using T5 − O1 and F4 − C4 channels.

Session	T5 − O1 channel					F4 − C4 channel				
	Precision (%)	Rate of accuracy (%)	Recall (%)	Overall amount of data	*F1*-score (%)	Precision (%)	Rate of accuracy (%)	Recall (%)	Overall amount of data	*F1*-score (%)
Usual EEG signal	79.18	89.35	86.01	152	82.91	70.18	74.62	90.01	152	72.91
Unusual EEG signal	82.12	81.6	71.43	127	75.92	83.12	82.98	56.43	127	65.32
Overall/avg.	80.65	85.48	78.72	279	79.42	76.65	80.65	78.2	279	69.12

**Table 5:** Comparison of existing mechanism and the proposed mechanism.

Method	Accuracy (%)	Precision (%)	Recall (%)	*F*1-score
Wavelet	82.53	81.6	83.46	—
DNN	74.63	77.08	73.10	73.09%
Proposed	85.48	76.65	78.2	69.12%

## Data Availability

The data used to support the findings of this study are included within the article. Further dataset or information is available from the corresponding author upon request.
